The article "A Feasible Multimodal Photoacoustic Imaging Approach for Evaluating the Clinical Symptoms of Inflammatory Arthritis" was retracted in 2023. Reasons: signs of a paper mill; compromised peer review; unreliable results or conclusions.

# A Feasible Multimodal Photoacoustic Imaging Approach for Evaluating the Clinical Symptoms of Inflammatory Arthritis

**DOI:** 10.1155/2022/7358575

**Published:** 2022-08-21

**Authors:** B. Rajasekar, P. Nirmala, P. Bhuvaneswari, R. Radhika, S. Asha, K. R. Kavitha, Semagn Shifere Belay

**Affiliations:** ^1^Department of Electronics and Communication Engineering, Sathyabama Institute of Science and Technology, Chennai, 600119 Tamil Nadu, India; ^2^Department of Electronics and Communication Engineering, Saveetha School of Engineering, SIMATS, Chennai, 602 105 Tamil Nadu, India; ^3^Department of Electronics and Communication Engineering, Sri Venkateswara College of Engineering and Technology, Chittoor, Andhra Pradesh 517127, India; ^4^Department of Electronics and Communication Engineering, S.A Engineering College, Chennai, 600077 Tamil Nadu, India; ^5^Department of Electronics and Communication Engineering, Saveetha Engineering College, Chennai, 602105 Tamil Nadu, India; ^6^Department of Electronics and Communication Engineering, Sona College of Technology, Salem, 636005 Tamil Nadu, India; ^7^School of Computing, Woldia Institute of Technology, Woldia University, Ethiopia

## Abstract

Numerous traditional medical imaging methods, including computed tomography with X-rays, positron emission tomography (PET), and magnetic resonance imaging (MRI), are utilized frequently in medical settings to screen for illnesses, diagnose patients, and track the effectiveness of treatments. When examining bone protrusions, CT is preferred over MRI for scanning connective tissue. Although the picture quality of PET is inferior to that of CT and MR, it is outstanding for detecting the molecular markers and metabolic functions of illnesses. To give high-resolution structural pictures and improved ailment sensitivity and specificity within another image, multimodal data and substantial therapeutic influence on advanced diagnostics and therapeutics have been used. The goal was to evaluate the clinical significance of multimodal photoacoustic/ultrasound (PA/US) articular imaging scoring, a cutting-edge image technique that may show the microvessels and oxygen levels of rheumatoid arthritis-related inflamed joints (RA). The PA/US imaging technology analyzed seven tiny joints. The PA and power Doppler (PD) impulses were semiquantified using a 0–3 grading scale, and the averages of the PA and PD scores for the seven joints are computed. Three PA+SO_2_ types were found determined by the relative oxygen levels (SO_2_) measurements of the affected joints. Researchers evaluated the relationships between the disease activity ratings and the PA/US imaging ratings. The PA scores and medical ratings that reflect the extent of the pain have strong relationships with each other, as do the PA+SO_2_ combinations. PA may be clinically useful in assessing RA. Thus, the research evaluated the clinical symptoms of inflammatory arthritis using a multimodal photoacoustic image process.

The article "A Feasible Multimodal Photoacoustic Imaging Approach for Evaluating the Clinical Symptoms of Inflammatory Arthritis" was retracted in 2023. Reasons: signs of a paper mill; compromised peer review; unreliable results or conclusions.

## 1. Introduction

Systemic autoimmune disorder rheumatoid arthritis (RA) is characterized by a continuous inflammatory illness, which damages joints and impairs functionality. The maximum speed of erosive joint illness occurs over the first two years, which is a proof that significant irreparable damage happens throughout this time frame, according to various researchers. In recent years, there has been mounting evidence that treatment intervention early in the RA disease phase results in previous disease management and fewer joint destruction. Furthermore, the evolution of potent and costly treatment medicines for RA has accelerated recently [1]. However, early arthritis is typically self-limiting in patients who are not already identified with RA. It is crucial to distinguish between RA and other types of arthritis as soon as symptoms appear because disease-modifying antirheumatic medications (DMARDs) for the prevention of a patient's arthritis are only warranted when these proportions are advantageous. RA must be viewed as a medical emergency requiring an immediate diagnosis and suitable care [2].

Due to its noninvasiveness and simplicity, Doppler US, especially color Doppler US (CDUS) and power Doppler US (PDUS), is frequently used to assess RA clinical symptoms and identify articular irritation. Regrettably, pathological alterations in the synovial membrane often manifest previously than favorable imaging assessment results. Additionally, latent inflammation, which manifests in arthralgia that is medically suspicious or in treatment outcomes following surgery, is probably not visible using standard scanning technology. In certain investigations, synovial biopsies have been used to identify the synovium's histologic and immunohistochemical (IHC) features for definitive diagnosis. Nevertheless, the invasive and labor-intensive synovial biopsy technique is only occasionally used [3]. To accurately and promptly diagnose synovitis in RA, innovative imaging techniques must be investigated. Some of the most recent imaging modalities built on the traditional US are contrast-enhanced US (CEUS) and photoacoustic imaging (PAI). Due to its low level of invasiveness and high expense, CEUS, in which gas-filled microbubbles (MBs) are injected as contrast media, has been extensively used in hospitals in Asia and Europe. By highlighting the expanded tiny capillaries in the inflammatory synovium, CEUS is useful in assessing arthritis. Additionally, MBs are a perfect vehicle for loading nucleotides, medicinal medicines, and antigens that has advanced molecular scanning and medicinal guiding. Additionally investigated in joint scanning is PAI, a brand-new noninvasive and nonionizing optical imaging technique [4].

The article "A Feasible Multimodal Photoacoustic Imaging Approach for Evaluating the Clinical Symptoms of Inflammatory Arthritis" was retracted in 2023. Reasons: signs of a paper mill; compromised peer review; unreliable results or conclusions.

Endogenous substances such as deoxyhemoglobin, collagen, lipids, oxyhemoglobin, and melanin enable OAI in the near-infrared (NIR) region because of their distinct absorption properties mentioned in Figure 1. The clinical utility of this method may eventually be enhanced by focused exogenous sensors or contrasting chemicals that precisely mark analytes or cells for further specialized imaging techniques. Due to the use of ultrasonic (US) vibrations, which reflect less in tissues than vision, OAI can recognize a wide variety of endogenous or exogenous chemicals within a unified imaging technique while preserving good spatial resolution at a larger depth than optical imaging. OAI can be widely applied in both clinical and experimental contexts without compromising biochemical functions because of its noninvasive character [5].

A major handicap is brought on by long-term active inflammatory arthritis, which also results in massive functional limitations, work loss, a lowered standard of living, and high medical expenses. Improving performance neuroimaging for early diagnostic and therapeutic result evaluation will be necessary for the creation of optimal and individualized therapy choices with potent new medications to stop the progression of the disease. As a result of their close relationship to the metabolism of inflammatory joint cartilage, physiologic variables like blood circulation, volume of blood, and plasma aeration could be crucial diagnostic indicators of arthritis. An important step in the chain of events leading to inflammation is the strong hyperemia of the afflicted joint, which results both from hypervascularization but also from dilation of the capillary network [6]. The inflammatory synovial membrane exhibits severe hypoxic, additional operational hallmark of inflammatory disease, as a result of the elevated metabolism of the swollen synovium as well as the comparatively insufficient oxygen supply of the inflamed joints. Recent research explores a connection between localized hypoxia within the synovial membrane of individuals having RA and inflammation-induced synovial fibroblast stimulation and enhanced tissue intrusiveness. Neoangiogenesis is induced by hypoxia, increasing the severity of synovitis, but the level of neoangiogenesis is uncertain to completely alleviate the hypoxia [7].

A rapidly developing biological imaging technique is photoacoustic (PA) image, commonly referred to as optoacoustic image analysis. The capacity of PA imaging to collect operational and biochemical data of actual time, having the higher spatial and temporal determination, at physiologically appropriate thicknesses, also without radiation exposure, may be its strongest point. Conventional imaging techniques do not offer the aforementioned balance of advantages. Endogenous contrasts in PA imaging could reveal operational and even anatomical features. Each one of these scanning approaches could be significantly improved by endogenous contrast media, which also enable imaging of molecular and cellular processes. These substances enable PA scanning to scan desired objects with respectable resolution and sensitivity. The capability of PA imagery as well as its implications increases with the sophistication of contrast media and molecular localization [8].

The article "A Feasible Multimodal Photoacoustic Imaging Approach for Evaluating the Clinical Symptoms of Inflammatory Arthritis" was retracted in 2023. Reasons: signs of a paper mill; compromised peer review; unreliable results or conclusions.

A new, nonionizing, noninvasive, reasonably priced method that can image both structurally and functionally is photoacoustic (PA) imaging (PAI). The architecture in living tissues that depend on optic contrasts could be traced at ultrasonic precision by first collecting the PA signals using US devices and then performing image reconstruction depending on the back-projection of the collected signals. In deeper, normal healthy finger joints, PAI has shown that it is capable of resolving the tissue structures using optic contrast and detecting inflammatory arthritis in animal studies. Real-time simultaneous PA and US scanning of a targeted joint has indeed been made possible by adding a laser pulse to a study US setup that is easily accessible and features a GPU card [9]. The possibility of real-time, low-cost dual-modality US and PA scanning of human finger joints utilizing a hand-held device combining a laser diode and transducer arrays coupled to a transportable US device has been investigated. A consumer-developed PA and US dual-modality setup utilizing concave arrays with great angular coverage was also used to obtain cross-sectional photography of a human finger. These dual-modality technologies might offer morphological and physiological data that are organically coregistered, and they might help with a thorough understanding of the pathogenesis in arthritic finger joints [10].

Spatial resolution is also impacted by scanning intensity. The majority of PA scanning, contrary to the microscope, is carried out at a depth exceeding 1 mm, in which the illumination is diffused. Given that diffused sunlight is distributed fairly uniformly, the properties of the US beam produced by a US transducer dictate the positioning accuracy in PA scanning. The transducer's frequency has an adverse relationship with axial (depth) accuracy. The image depths, as well as the center frequency and shape of the US transducers, all influence the resolving power. The best resolution scans are performed by transducers with a high center frequency bandwidth. For instance, it is possible to attain axial frequencies of 15 and 150 *μ*m and laterally resolution of 50 and 300 *μ*m utilizing 50 MHz and 5 MHz transducers, correspondingly. If the illumination is properly concentrated within the tissues and photography is limited to the ballistic domain of incident light, often within or less than 1 mm thickness, PA scanning could attain even higher horizontal resolution (5 *μ*m). The high-frequency components of the pressure change are preferentially muted as it proceeds through the tissues and drifts away from the photo absorber. As a consequence, the PA transmitter range and center frequency are reduced. Consequently, as imaging depths rise, the spatial resolution must diminish over time [5].

The article "A Feasible Multimodal Photoacoustic Imaging Approach for Evaluating the Clinical Symptoms of Inflammatory Arthritis" was retracted in 2023. Reasons: signs of a paper mill; compromised peer review; unreliable results or conclusions.

Over the past ten years, PAI, which is dependent on the photoacoustic (PA) impact, has received more attention in biomedical activities. Molecular contrasts of absorption spectra are provided by PAI, which makes use of the deep imaging capabilities of ultrasonic imaging. The optical excitation and ultrasound (US) monitoring processes form the foundation of the PA effect. During the optic stimulation stage, biological structures are illuminated by a burst of light, which is then collected by scanning objectives. As the item expands and contracts as a result of the heat created by the light absorption, the target inside the item releases acoustic waves (US). Acoustic waves travel through the material during the US identification process and are detected by a traditional US transducer to produce images with just an absorption spectrum difference [11]. The benefits of traditional USI could be transferred directly to PAI thanks to the organic integration of sound and light. Because PAI combines the morphology picture of USI with the functional image of PAI, it is intrinsically a multimodal imaging technique. A wide range of multiresolution PAI devices, including tomography and microscopy structures, have already been researched in the research. In 10 RA patients with medically obvious synovitis, elevated PA values were found by a transportable PA/US imaging instrument and had a good connection with PDUS, as per the research. Although there has not been a thorough comparison among PA/US scanning and clinical techniques of RA assessment, the larger samples of the earlier research were generally modest. More research concentrating on the clinical assessment and verification of PAI is required to better investigate the clinical uses and utility of PAI in RA [12].

The article "A Feasible Multimodal Photoacoustic Imaging Approach for Evaluating the Clinical Symptoms of Inflammatory Arthritis" was retracted in 2023. Reasons: signs of a paper mill; compromised peer review; unreliable results or conclusions.

In this work, researchers used a multimodal PA/US imaging technology, which combines a light source with an ultrasonic transducer, to image the joints of RA patients. Researchers sought to determine the relationship between the relative oxygen saturation (SO2) levels of lesion on multifunctional PA/US articular imaging and various RA symptomatic parameters, as well as the possible benefits of multimodality PA/US screening of RA in clinical practice.

## 2. Related Works

Anterior cruciate ligaments are the human body's most frequently injured ligaments (ACLs). ACL injuries are common among athletes who play basketball, football, and soccer. With the aid of effective and extensive automated magnetic resonance and a DL approach, the study was aimed at examining anterior cruciate damage at a preliminary phase. The method put forward in this study made use of class balance and data enrichment to create a modified 14-layer ResNet-14 convolutional neural network (CNN) with six various directions. Utilizing the modified ResNet-14 DL architecture with a combination category proper balance and real-time data strengthening, the performance was assessed using specificity, precision, sensitivity, accuracy, and F1 score. The results were 0.920 percent, 0.916 percent, 0.946 percent, 0.916 percent, and 0.923 percent, respectively. The area under curves (AUCs) for healthy tear, partial tear, and fully ruptured break for the suggested ResNet-14 CNN were correspondingly 0.980 percent, 0.970 percent, and 0.999 percent. According to the provided diagnostic testing, this method is utilized towards predicting automatic identification and assessment ACL injuries in sportsmen using the suggested deep learning methodology. There are several limitations that have been identified in this research; ResNet-14 model for ACL tear detection worked independently on each of the six methods, which can add to the overall training load. The method was also applied to hybrid class balancing, which arbitrarily improved the records in the partially ruptured and fully ruptured tears. It was not a good idea to downsample the class label of healthy ACLs in the metadata file since this could have affected the results in the case of the entirely ruptured class. Future research that employs class loading would see an even greater improvement in the ACL tear-detecting system's efficiency. Additionally, given the absence of class balance, the findings were not tested using more than 5-fold cross-validation [13].

Rheumatoid arthritis commonly manifests as cervical spine lesions (RA). This research's objective was to retrospectively analyze radiology abnormalities in the spinal cord within RA patients and connect the results with clinical and biochemical data. Clinicians submitted 240 RA cases in a row for neuroimaging as a result of complaints that suggested cervical spine degeneration and/or a protracted illness course. Each patient had lateral radiography taken as well as a cervical spine magnetic resonance. Testing results and screening patients were linked with the images acquired. In 179 cases, the cervical spine was impacted. Subaxial subluxation, anterior atlantoaxial subluxation, and demineralization were the most frequent lesions. Basilar settlement (*p* = 0.003), subaxial subluxation (*p* = 0.005), and posterior AAS (*p* = 0.005) were all linked to prolonged duration of illness. Up to 75% of RA patients experience the development of lesions which can be seen in magnetic resonance imaging and radiography. The front AAS and subaxial subluxation are the radiographic abnormalities that are most frequently observed. Risk variables for spinal cord participation included long illness history, RF seropositivity, and elevated inflammatory biomarkers. The primary drawback of radiography is the obscuration of anatomic structures caused by the superimposition of morphological characteristics utilized as measuring points of reference [14].

The article "A Feasible Multimodal Photoacoustic Imaging Approach for Evaluating the Clinical Symptoms of Inflammatory Arthritis" was retracted in 2023. Reasons: signs of a paper mill; compromised peer review; unreliable results or conclusions.

Minimal data about the prevalence of the illness is presented in a recent analysis of thermography investigations in rheumatoid arthritis, which also highlights the discrepancies between the thermography of people with Alzheimer's disease and that of healthy individuals. A retrospective analysis that considered demographics, medical, laboratory, and temperature measurement factors contrasted people with elevated disease severity, moderate clinical symptoms, and healthy individuals. Researchers used a finger inspection methodology and an infrared thermal imaging device. The results have the average temperature of five fingers of a hand in stationary, postcooling, and post-rewarming, as well as the complete change in a temperature increase of fingers caused by cold incitement and the massive modification in mean temperature of fingers due to reheating. Other results have included the area underneath the cooling and heating curvatures, the distinction between the two, and temperature intensity distribution charts. In proportion of patients with medium disease severity, individuals with elevated disease severity had a narrower range under the heating cycle, a smaller comparison among the area underneath the process gradually curves and the cooling bend, and a slightly smaller increase in average temperatures due to rewarming (*p* > 0.05). The article's drawback is the dearth of prospectively examined members of the groups with mild clinical symptoms. The interpretation of the results must be viewed as exploratory with this cohort. For more accurate information, further research and individuals are required. These outcomes need to be confirmed in additional research to be useful to individuals with minimal clinical symptoms [15].

The article "A Feasible Multimodal Photoacoustic Imaging Approach for Evaluating the Clinical Symptoms of Inflammatory Arthritis" was retracted in 2023. Reasons: signs of a paper mill; compromised peer review; unreliable results or conclusions.

Rheumatoid arthritis (RA) is an autoimmune disorder that has systematic, persistent, and inflammation consequences on the musculoskeletal. The condition frequently progresses, impairs physical ability, results in pain and exhaustion, and damages the joints. Over time, RA damages the cartilage and bone in the joint, affects the tendons and ligaments surrounding the joints, and ultimately resulted in joint damage. It is common to practice gathering information for RA using devices, which includes accelerometers, wearable sensors, and thermal infrared camera sensors. This research discusses the categorization of medical illnesses based on databases from RA and orthopedics utilizing ensemble approaches. The RA database was collected by the assessment of white blood cell categorization utilizing attributes taken from a digital microscopy image of lymphocytes. The study included three ensemble methodologies: Adaboost, bagging, and random segmentation. As the basis for learning for the ensemble classifiers, k-NN (k-nearest neighbors) and random forest (RF) are being used. Utilizing holdout and 10-fold cross-validation assessment processes, the data analysis is obtained. The evaluation was based on a combination of performance metrics, including the receiver operating characteristic (ROC) curve, F-measure, accuracy, and recall. Additionally, the total classifier efficiency rate across various ensemble classifiers and the base learners was compared to evaluate performance. In general, it was discovered that bagging-RF exhibits the highest total average accuracy of 94.84 percent among several ensemble classifiers for dataset 2, while the random subspace classifier with k-NN exhibits the best outcomes for dataset 1 in terms of overall average accuracy of 97.50 percent. The results show that the basic classifiers' effectiveness with the various classifiers has significantly increased. The machine learning community mostly researched ensembles of weak learners [16].

Three-dimensional (3D) images, such as those produced by computed tomography (CT) and magnetic resonance imaging, are frequently employed in the medical field (MRI). The 3-dimensional MRI is a noninvasive technique for researching osteoarthritis in the soft tissue components of a knee joint. By determining the bone structure first, it can significantly increase the precision of segregating tissues including cartilage, bone marrow lesions, and meniscus. A convolutional neural network called U-net was created to segment biological images using less data for training. A single 2D image serves as the original U-input net, while a binary 2D image serves as the outcome. In this research, researchers altered the U-net model to recognize the knee bony protrusions from a series of 2D slices taken during 3D MRI. The detection and segmentation of knee bones have been suggested using a fully automatic approach. With 99 knee magnetic resonance instances, every instance has 160 2D segments for a single knee scan; the developed framework was trained, evaluated, and verified using these data. The identity, dice coefficient (DICE), and area error metrics were computed to assess the effectiveness of the system. The tibia, femur, patella, and a composite framework for fragmenting all the knee bones were used in independent factors that were trained. The approach was able to determine the beginning and ending bones slicing utilizing the entire MRI sequence (160 slices) and then divide the denser bones for all subsequent slices. The segmentation model obtained DICE 96.94 percent and similarities 93.98 percent on the testing set, while the detection model scored 98.79 overall accuracies. In terms of DICE scores utilizing the same database, the suggested method outperforms numerous state-of-the-art methods, including U-net, SegNet, and FCN-8, by a combined 3.68 percent, 14.45 percent, and 2.34 percent. There are a few restrictions on this research. The little dataset comes first. For segment jobs, data labeling takes a long time, particularly when delineating the various bone sections manually for 3D MRI image series. This made it impossible for us to include more information in this analysis. Researchers intend to use unsupervised learning or semisupervised learning in the future by making handling huge databases easier [17].

The article "A Feasible Multimodal Photoacoustic Imaging Approach for Evaluating the Clinical Symptoms of Inflammatory Arthritis" was retracted in 2023. Reasons: signs of a paper mill; compromised peer review; unreliable results or conclusions.

## 3. Methodology

### 3.1. Basic PA Imaging

Essentially, the PA impact is the creation of auditory waves as an outcome of optical light absorbing. While numerous processes could result in the formation of a PA indication, thermoelastic tissue displacement is what is used in biological PA scanning. The tissue is exposed to a pulsed laser beam for a nanosecond during PA scanning. Endogenous chlorophylls, such as melanin or hemoglobin, or exogenous contrasting materials, such as chemicals or nanomaterials, soak up the energy from the sun and transform it into heat. The tissue experiences rapid thermoelastic extension as a result of the heat. A broadband compression waveform that starts from the photo absorber is then produced by the tissues [18]. A standard ultrasound (US) receiver may identify this pressure gradient. The definition of the greatest starting pressure, *P*^0^, produced by the absorbers is presented in

(1) $$\begin{array}{c} P^{0}=\Gamma \delta_{a}F, \end{array}$$

where Γ is the tissue's Gruneisen variable, *F* is the light's fluency at the photo absorber, and *δ*_*a*_ is the photoabsorber's absorption spectrum efficiency. Only the PA pressure strength at the absorbent is predicted by this equation. In reality, the pressure waves produced by the incoming laser energy will be diminished in the tissues (through optic and acoustical absorption and scattering); this reduction depends on the different wavelengths and US frequencies. Penetration depth is the primary factor limiting the range of PA scanning. Safe laser exposure limits (20-100 mJ/cm^2^ for human skin contact to a laser pulse working at comparable optical different wavelengths from 400 to 1500 nm) were used to achieve thicknesses of up to 5–6 cm [19]. This stated depth works significantly better than ballistic optical imaging techniques, such as optical coherence tomography (OCT), which are only capable of reaching depths of about 1 mm. Resolution is also impacted by scanning intensity. The majority of PA imaging, contrary to the microscope, is carried out at depths exceeding 1 mm, where the illumination is diffused. Given that dispersed lighting is distributed fairly uniformly, the properties of the US beam produced by a US transducer dictate the spatial resolution in PA scanning. The transducer's bandwidth has an adverse relationship with axial (depth) accuracy. The imaging depth, as well as the frequency band and shape of the US transducers, all influences the resolving power. The best resolution images are generated by transducers with a high center frequency bandwidth. For instance, it is possible to attain an axial resolution of 15 and 150 *μ*m and horizontal frequencies of 50 and 300 *μ*m utilizing 50 MHz and 5 MHz transducers, correspondingly [20].

If the light is precisely concentrated in the tissues and scanning is limited to the kinetic phase of waveguides, often within just under 1 mm thickness, PA scanning could attain even higher lateral resolutions (5 *μ*m). The frequency components of the pressure change are preferentially muted as it passes through tissues and drifts away from the photo absorber. As an outcome, the PA signal's bandwidth and center frequencies are reduced. As scanning thickness grows, the resolution must always decrease. In PA imaging, optical absorption provides the primary contrast. Therefore, imaging endogenous chromophores like hemoglobin, melanin, and lipids are a good application for PA imaging. These chromophores exhibit large wavelength-dependent variations in their optical absorption. Consequently, distinct absorbers could be identified using spectroscopic techniques. The imaging of blood arteries, measurement of oxygen levels, identification of melanoma, and detection of lipids in vessels have all been accomplished using spectroscopy PA (sPA) [21].

The article "A Feasible Multimodal Photoacoustic Imaging Approach for Evaluating the Clinical Symptoms of Inflammatory Arthritis" was retracted in 2023. Reasons: signs of a paper mill; compromised peer review; unreliable results or conclusions.

### 3.2. Data Collection

A cross-sectional strategy was used for creating this research. The Peking Union Medical College Hospital's (PUMCH) Institutional Review Board gave its permission to every step of this research's operations (approval number: JS-1923). All participants who were recruited provided written, fully informed permission. In between December 2018 and October 2019, RA sufferer elder than 18 has been sought out at PUMCH's rheumatic outpatient department. As per the 2010 American College of Rheumatology/European League against Rheumatism (ACR/EULAR) categorization standards, the cases were treated with RA. Individuals with difficult cases of other forms of arthritis, such as OA, ReA, and gouty joint problems, were not included [22].

### 3.3. Multimodal PA/US Imaging System

Figure 2 displays the dual-modality imaging system's block diagram. As the primary platform for this innovative camera system, available commercially ultrasonic technology outfitted with an OPO potentiometer light and a hand-held linear probe centered at 5.8 MHz was used. The PA imaging option can show PDUS and grayscale US (GSUS) together instantaneously. For PAI, the wavelength at which poorly absorbed hemoglobin and oxygenated hemoglobin might reach their relative maximal absorption levels is 750 nm and 830 nm. The technology supplied synchronized grayscale US and 830 nm PAI at a frame rate of 10 Hz [23].

The accompanying scanning parameters were used for power Doppler US: a rectangular sampling box with no angulation, a high pulse rate of 600–1000 Hz, a wall filter of 50–100 Hz, a maximum intensity of 85–90%, and a scale of 3 cm/s.

### 3.4. Photoacoustic Imaging

One of the biological imaging techniques with the fastest growth is photoacoustic scanning. The model is founded on Bell's discovery of the photothermal phenomenon in 1880. Typically, after being exposed to brief laser beams, the intensity of the photon is absorbed by exogenous or endogenous chromophores within the tissues. This energy absorption then causes a brief local temperature increase, which then, in turn, can cause thermoelastic contraction to produce pulses. An acoustic detector could record these changes in pressure, which travel through tissues as ultrasonic waves and turn them into the image of the dispersion of the chromophore within the material [24]. The carrier frequency of produced ultrasonic signals may reach many tens or hundreds of megahertz, dependent on the spatial sizes of the optic absorber. The PA production procedure has no bearing on the signal's frequency or equivalent spatial and temporal resolution. Conversely, the highest observed frequency of the PA pulse is constrained and, consequently, dictates the feasible pixel density due to the frequency-dependent acoustical absorption occurring in tendons. The resolution in PAI, therefore, increases with distance. The spatial resolution of PAI systems may also be constrained by the ultrasonic detector's characteristics, such as its frequency, central wavelength, design variables, and detecting apertures.

The article "A Feasible Multimodal Photoacoustic Imaging Approach for Evaluating the Clinical Symptoms of Inflammatory Arthritis" was retracted in 2023. Reasons: signs of a paper mill; compromised peer review; unreliable results or conclusions.

Both photoacoustic tomography (PAT), which employs a reconstruction-based interference pattern, and photoacoustic microscope (PAM), which uses a focused-based interference pattern, can be classified as PAI. Typically, a widefield misdirected stimulation light and an array of the ultrasonic detector are employed in photoacoustic scanning to concurrently analyze the produced ultrasonic wave at numerous locations [25]. It has been utilized in various applications including new treatments and whole-body scanning of tiny animals because it can produce scans with a wide view. PAM, as opposed to PAT, relies on raster-scanning of optic and acoustic focuses and creates image files from captured depth-resolved information. PAM is typically the option of choice for use in situations that favor better resolution above the extensive depth of penetration, such as single-cell scanning. PAM could be further broken down into optical-resolution PAM (OR-PAM), in which the optical concentrating prevails the quality, and acoustic-resolution PAM (AR-PAM), where the acoustic concentrating is tighter than optically focused. The scanning arrangement for various photoacoustic scanning configuration options is shown in Figure 3. According to the deployment, photoacoustic endoscopy (PAE), which will be used to image inside tissue or organs, could be regarded as a subclass both of PAM and PAT. PAE typically offers micron-scale spatial resolution and millimeter-scale scanning depth [11].

The integration of optical radiation and acoustic recognition in photoacoustic scanning devices results in two different benefits. Initially, they offer the special absorption spectrum diagnostic difference. As a consequence, PAI allows maximum sensitivity identification of endogenous chromophores such as lipids, melanin, hemoglobin, collagen, and cytochrome that are moderately fluorescent and challenging or impracticable to identify with external fluorophores. This supports current dominant in vivo optically molecular scanning technologies, such as fluorescence microscopy, which is a recognized imaging technology. Secondly, PAI allows for a broad scaling range of spatial and temporal resolution and penetrating levels beyond substantial (i.e., 100–400 m accuracy at the thickness of many centimeters) [26]. The modalities are an effective tool for biology and medicine because it also offers order to better facilitate chemical imaging characteristics. Photoacoustic spectroscopic, which relies on the capacity to selectively photograph particular chromophores by adjusting the emission spectrum, is another one of those well-known skills. Thus, the number of particular chromophores could be measured using spectroscopic research and the acquisition of pictures at various wavelengths. For instance, the absorbance spectrum of plasma at transparent and near-infrared wavelengths is strongly influenced by its oxygen saturation (SO_2_) and, as a result, by the stark spectral contrast between oxyhemoglobin (HbO_2_) and deoxyhemoglobin. This spectrum differential can be used to measure SO_2_, a significant physiological variable associated with several pathological conditions and inflammatory conditions, as well as measure the levels of HbO_2_ and HHb. Doppler flowmetry and photoacoustic pioneering work, two more functional expansions of PAI, have made it possible to assess blood circulation velocities and acquire maps of temperature profiles in tissue, accordingly [27].

The article "A Feasible Multimodal Photoacoustic Imaging Approach for Evaluating the Clinical Symptoms of Inflammatory Arthritis" was retracted in 2023. Reasons: signs of a paper mill; compromised peer review; unreliable results or conclusions.

Because of the distinctive and significant imaging benefits that PAI provides, it is the modality of choice for a wide range of functional and biochemical sensing applications. It is being used in a wide range of clinical and preclinical implementations, such as image analysis of blood oxygen levels, image processing of the brain's vascular system and feature, imaging of the expression of genes, diagnosing defenseless atheromatous inscriptions, image processing of skin malignant tumors, scanning of histology-like tissues, longitudinal tumor angiogenesis research, imaging and recognition of protein complexes, and imaging of synthetic biology formwork.

### 3.5. Imaging Protocols

The study's seven-joint ultrasonic score scheme (US7) was used as a guide to select joints for the multimodal PA/US exams. Multimodal scans were performed on the medically dominant side at the 3rd metacarpophalangeal joint (MCP3), 3rd proximal interphalangeal joint (PIP3), 2nd proximal interphalangeal joint (PIP2), 2nd metacarpophalangeal joint (MCP2), 2nd metatarsophalangeal joint (MTP2), 5th metatarsophalangeal joint (MTP5), and wrist. A US operator with one year of musculoskeletal US expertise and one month of model development performed real-time PA/US scanning after performing GSUS and PDUS scanning of the joints [20].

The article "A Feasible Multimodal Photoacoustic Imaging Approach for Evaluating the Clinical Symptoms of Inflammatory Arthritis" was retracted in 2023. Reasons: signs of a paper mill; compromised peer review; unreliable results or conclusions.

### 3.6. Semiquantitative PDUS and PAI Scoring

To evaluate PD and PA photos in the research, the semiquantitative point's structure graded around the range of 0–3 suggested for PDUS has been used as a basis. For data analysis, the combined PDUS (PD sum, 0-21) and PA (PA sum, 0-21) values 7 bones have been computed. Multiple radiologists having two years of collective expertise in the musculoskeletal US evaluated the images without knowing the identities of the individuals or the clinical features of the joints being looked at. Reconfirmations of the photographs were done when there were disagreements until an agreement was obtained. The two raters evaluated the PD and PA photos once more after a week. Both raters evaluated the PD and PA photographs once again after one week: intraobserver consensus of the two rating sessions and interobserver concordance of the first standard session between the two reviewers.

### 3.7. Sulphur Dioxide and PA+Sulphur Dioxide Analysis Pattern

The relative SO_2_ levels of the inflamed tissue were calculated by dividing the pixel of the PA readings in the target regions at a wavelength of 750 nm and 830 nm. Based on the dispersion of the relative SO_2_ levels, the participants were separated into categories of hyperoxic and hypoxic conditions. After computing the sulphur dioxide readings, the sulphur dioxide score and the PA sum rating were combined to create the “PA+SO_2_ patterns,” a novel index for RA patients. Individuals with PA sum values below three were thought to have only weak PA signals, whereas those with PA scores above three were thought to have strong PA signals. Each individual was assigned to one of three groups based on their SO_2_ levels and PA sum goals scored: pattern 1 (no or minimum PA signals), pattern 2 (obvious PA signals and hyperoxia), and pattern 3 (evident PA signals and hypoxia). Additionally, assessed were the relationships between the medical ratings and the PA+SO_2_ patterns [13].

### 3.8. Assessment

Age, sex, disease length from the start and diagnostic verification, period of pain and stiffness, symptomatology, and medication lists were all noted along with other pertinent patient data. Erythrocyte sedimentation rate (ESR), anti-cyclic citrullinated peptide (anti-CCP) antibodies, C-reactive protein (CRP), and inflammatory antigen were among the scientific measurements taken from the patients (RF). A rheumatologist with 18 years of expertise in medical rheumatism evaluated 28 joints for swelling and sensitivity (the swollen joint count (SJC) and the tender joint count (TJC)) for each patient. These joints included wrists, bilateral PIPs, elbows, shoulders, MCPs, and knees. Joint pain visual analog scale (VAS) ratings, as well as data for the severe clinical activity index (CDAI), simplified disease activity index (SDAI), disease activity score in 28 joints (DAS28), and patient global activity (PGA) were also obtained.

The article "A Feasible Multimodal Photoacoustic Imaging Approach for Evaluating the Clinical Symptoms of Inflammatory Arthritis" was retracted in 2023. Reasons: signs of a paper mill; compromised peer review; unreliable results or conclusions.

### 3.9. Statistical Analysis

Controlled rates, such as imaging results, clinical results, and laboratory results, are described using the average as well as standard deviation (SD). Spearman's rank correlation value was used to assess associations among imaging ratings (PA sum rates, PD sum scores, and the three PA+SO_2_ patterns) also the clinical rankings. Patterns 1, 2, and 3 of the PA+SO_2_ are viewed as ordinal categorical data. The following was the interpretation of the coefficient of correlation: low positive correlation is 0.31 to 0.51, moderate positive correlation is 0.51 < *ρ* < 0.71, high correlation is 0.71 < *ρ* < 0.91, and very high positive correlation is *ρ* > 0.91. The weighted kappa value, which is provided with a 95% confidence interval, was used to assess the intraobserver and interobserver agreement between two radiologists (97 percent CI) [25]. The following explanation applied to the value: poor: *μ* < 0.21, impartial: *μ* < 0.21, reasonable: *μ* < 0.41, finest: *μ* < 0.62, enormously finest: *μ* < 0.81, and very good: *μ* < 1.00. For statistical analysis, SPSS software (version 21.1) was utilized. The weighted kappa value, which is provided with a 97 percent confidence level, was used to assess the intraobserver and interobserver agreement between two radiologists (97 percent CI). The following explanation applied to the value: poor: *μ* < 0.21, impartial: *μ* < 0.21, reasonable: *μ* < 0.41, good: *μ* < 0.61, enormously finest: *μ* < 0.81, and very good: *μ* < 1.00. For numerical examination, SPSS software has been utilized [10].

## 4. Result and Discussion

For this trial, the overall of 31 RA patients would be included, comprising 24 females and 7 males between the ages of 25 and 71 (mean age 51.9, median age 52). The PA/US method was used to examine 217 bones' totality.  Table 1 provides an overview of the patients' complete clinical evidence. The intraobserver consistency for rater 1 is 0.87 (0.76-0.96) for two PD scores (*p* = 0.042) and 0.89 (0.80-0.95) for 2 PA scores (*p* = 0.044). The intraobserver consistency for rater 2 was 0.93 (0.85-1.00) for PD assessment and also 0.89 (0.82–0.98) for PA scoring, correspondingly (*p* = 0.044 and 0.046). Most evaluators had excellent intraobserver consistency when grading the PD and PA photos.

The article "A Feasible Multimodal Photoacoustic Imaging Approach for Evaluating the Clinical Symptoms of Inflammatory Arthritis" was retracted in 2023. Reasons: signs of a paper mill; compromised peer review; unreliable results or conclusions.

Additionally, the two physicians' interobserver concordance for rating the pictures was excellent (=0.84 (0.74-0.93) with PD rating and 0.83 for PA rating (*p* = 0.046)). The PA/US method was used to analyze 217 joints in total, and Table 2 lists the numbers for each PA grade and the matching PD grade (0-3) for each joint. 16 joints, out of all those tiny joints, were classified as having the greatest PA as well as PD levels. It has 21 joints with level 1 PA scores that does not have PD indications.

RA disease activity analysis is based on correlation between PA/PD.

Table 3 shows the correlation between the B-PA sum scores, A-PD sum scores, and RA infection activity measurement. The B-PA sum had strong positive correlations with the DAS28 (ESR) (*ρ* = 0.755 (0.547-0.876), *p* < 0.0002), DAS28 (CRP) (*ρ* = 0.797 (0.616-0.898), *p* < 0.0002), SDAI (*ρ* = 0.837 (0.685-0.9189), *p* < 0.0002), and CDAI (*ρ* = 0.838 (0.688-0.918), *p* < 0.0002) High positive correlations between the PA sum and TJC and SJC were observed (*ρ* = 0.802 (0.621-0.902), *p* < 0.0002 and *ρ* = 0.793 (0.605-0.897), *p* < 0.0002, correspondingly). The associations between the PD sum and the TJC and SJC ranged from medium to high (*ρ* = 0.718 (0.485-0.858), *p* < 0.0002 and *ρ* = 0.698 (0.454-0.847), *p* < 0.0002, correspondingly). The A-PD sum had a mild positive association with CRP (*ρ* = 0.433 (0.0923-0.683), *p* = 0.0152), whereas the PA sum had a moderately positive connection (*ρ* = 0.545 (0.236-0.754), *p* = 0.0017).

The PD sum and PA sum did not interact with ESR. The coefficient value between the PA sum ratings and the patient's VAS pain rating was significant (*ρ* = 0.699 (0.452-0.847), *p* < 0.0002), and it was greater than A-PD sum (*ρ* = 0.509 (0.182-0.735), *p* = 0.0042). While the PD sum scores were unrelated to the global evaluation (PGA = 0.483 (0.148-0.719), pv = 0.0071), the B-PA sum has a modest connection in it.  Figure 4 displays the fitting lines for the clinical ratings and PD/PA rating findings. Each curve showed an increasing trend, confirming the links between the radiological and detection of the disease.

Relative sulphur dioxide levels were determined for 21 of the 31 patients who had visible PA signs. The 10 instances with a PA sum of 0 and no discernible PA impulses within inflammatory cells were disregarded for measuring sulphur dioxide. The tiny joints' sulphur dioxide level was 87.6 ± 10.2 percent. As per the pattern of the absolute sulphur dioxide values, the individuals were split into the hypoxic and hyperoxic subgroups. Nine cases were classed as hypoxic, with a comparative sulphur dioxide value of less than 85%, while twelve individuals were categorized as hyperoxic, with a value higher than 91%.

The article "A Feasible Multimodal Photoacoustic Imaging Approach for Evaluating the Clinical Symptoms of Inflammatory Arthritis" was retracted in 2023. Reasons: signs of a paper mill; compromised peer review; unreliable results or conclusions.

Table 4 displays the clinical ratings for the three patterns. Substantial variations among individuals with obvious PA indications and those that were labeled as hypoxic and hyperoxic were found in the VAS paining rate and PGA (patterns 2 and 3). The other indices showed no patient-specific variations.  Figure 5 shows a strong positive association between the PA+SO^2^ patterns and the VAS pain score.

In this research, the minor bones of RA patients with a variety of disease severity were assessed using a composite PA/US imaging technology. The diagnostic ratings and the PA characteristics, such as the PA sum score and PA+SO_2_ sequences, had strong correlations, indicating the viability of using PAI to measure the clinical symptoms of RA. PAI may be used as methods and technologies associated with US also to standard grayscale US as well as PDUS to just provide fresh imaging data to aid in determining the disease activity of RA. Utilizing a 0–3 PDUS leveling system as well as the condensed US7 points system as a guide, we performed a comprehensive radiological evaluation of minor joints in RA patients, such as the MCP, PIP, MTP, and wrist.

Implying that the PAI is just more susceptible to tiny vasculature within the hypertrophied synovium and inflammatory tendon sheathing than PDI, the PA sum rates of the seven bones have highest value than PD sum values. Abundant PA impulses were also visible in tumors with the greatest PD score, 3, which is the highest mark. Evident PA signals were observed in some joints for the synovial hypertrophic places with low PD scores, such as 0 and 1, suggesting certain RA instances, dynamic inflammatory which might be seen on PAI assessments or might not be seen on traditional US exams. This study found a medium to a high association between the PD ratings and clinical scores, with a regression analysis of 0.40 to 0.72. This outcome was in line with the ratio of 0.47 to 0.64 from earlier investigations. The PA sum number exhibited a greater coefficient of correlation than the PD sum rating, and it showed a strong positive connection through common medical infection ratings. Consequently, PAI can precisely represent each patient's progression of the disease, which is especially beneficial for aggressive lesions that are challenging for PDUS to detect.

## 5. Conclusion

There are links between the PA ratings of the microvasculature and the clinical features ratings for RA, and there is also a relationship between comparative SO_2_ and the diagnostic ratings that indicate the intensity of the pain. The multifunctional PA/US imaging technology offered thorough imaging characteristics and may hold significant promise in the assessment of RA patients' disease severity. The relevance of SO_2_ in the diagnosis of RA is also anticipated to be investigated in future clinical research with larger samples. Secondly, prospective longitudinal research will need to be conducted in the approach to see whether the PA measurements in this study could forecast response to therapy and the risk of RA relapse. This work is the first cross-sectional observational analysis using multifunctional PA/US image acquisition.

The article "A Feasible Multimodal Photoacoustic Imaging Approach for Evaluating the Clinical Symptoms of Inflammatory Arthritis" was retracted in 2023. Reasons: signs of a paper mill; compromised peer review; unreliable results or conclusions.

## Figures and Tables

**Figure 1:** Different optoacoustic imaging molecule and tissues.

**Figure 2:** Block diagram of PA/US system.

**Figure 3:** Generation and detection based on signal.

**Figure 4:** Image scoring fitting curve and scatter points.

**Figure 5:** Clinical score fitting and scatter points (VAS and PGA).

**Table 1:** Medical features of RA patients.

Features	Average value
Age	51.9 ± 12.4
Erythrocyte sedimentation	21.5 ± 26.3
C-reactive protein	12.4 ± 24.6
Inflamed jt counts	7.6 ± 8.1
Tender jt counts	7.3 ± 8.2
Pain visual analog scale	24.4 ± 3.13
Patient global activity	26.6 ± 30
Evaluator global activity	22.5 ± 26.6
Infection rate in 28 joints (CRP)	3.8 ± 2.2
Infection rate in 28 joints (ESR)	3.8 ± 1.1
Simplified disease index	21.2 ± 20.2
Medical infection index	19.5 ± 19
PD sum of power	2.9 ± 3.4
PA sum of power	4.6 ± 3.8

**Table 2:** PD score and PA.

Photoacoustic score	Power Doppler score				Overall
	A	B	C	D	
A	148	0	0	0	148
B	22	5	0	0	27
C	6	3	11	0	20
D	0	3	5	14	22
Overall	176	11	16	14	217

**Table 3:** RA infection and correlation coefficient of A-PD and B-PA.

		Correlation coefficient	97% confidence interval	Probability rate
Erythrocyte sedimentation	A-PD sum	0.212	-0.155-0.527	0.255
	B-PA sum	0.26	-0.0993-0.567	0.263
C-reactive protein	A-PD sum	0.433	0.0923-0.683	0.0152
	B-PA sum	0.545	0.236-0.754	0.0017
Swollen joint count	A-PD sum	0.700	0.454-0.847	<0.0002
	B-PA sum	0.793	0.505-0.97	<0.0002
Tender joint count	A-PD sum	0.720	0.485-0.858	<0.0002
	B-PA sum	0.802	0.621-0.802	<0.0002
Paining visual analog scale	A-PD sum	0.509	0.182-0.735	0.0032
	B-PA sum	0.699	0.452-0.845	<0.0002
Patient global activity	A-PD sum	0.197	-0.177-0.521	0.299
	B-PA sum	0.483	0.148-0.719	0.0071
Evaluator global activity	A-PD sum	0.422	0.0713-0.679	0.0205
	B-PA sum	0.623	0.339-0.804	0.0023
Disease activity score in 28 joints (CRP)	A-PD sum	0.652	0.386-0.818	0.0002
	B-PA sum	0.755	0.547-0.876	<0.0002
Disease activity score in 28 joints (ESR)	A-PD sum	0.677	0.423-0.832	<0.0002
	B-PA sum	0.797	0.616-0.898	<0.0002
Simplified disease activity index	A-PD sum	0.717	0.485-0.855	<0.0002
	B-PA sum	0.837	0.685-0.919	<0.0002
Clinical disease activity index	A-PD sum	0.710	0.474-0.851	<0.0002
	B-PA sum	0.838	0.690-0.920	<0.0002

The article "A Feasible Multimodal Photoacoustic Imaging Approach for Evaluating the Clinical Symptoms of Inflammatory Arthritis" was retracted in 2023. Reasons: signs of a paper mill; compromised peer review; unreliable results or conclusions.

**Table 4:** PA+SO_2_ pattern of clinical scores.

	Pattern 1 (*n* = 10)	Pattern 2 (*n* = 12)	Pattern 3 (*n* = 9)	*p* value^∗^	*p* value^∗∗^
Erythrocyte sedimentation rate	13.9 ± 14.5	26.9 ± 32.1	26.6 ± 30.5	0.3307	0.607
Simplified disease activity index	3.5 ± 2.9	24.7 ± 15.9	39.4 ± 21.7	<0.002	0.085
Clinical disease activity index	3.4 ± 2.5	22.9 ± 13.7	36.9 ± 20.5	<0.002	0.068
C-reactive protein	3.6 ± 5.7	17.6 ± 36.5	19.4 ± 19.5	<0.002	0.959
Infection rate in 28 joints (ESR)	1.8 ± 2.0	5.5 ± 2.6	6.3 ± 2.5	<0.002	0.354
Infection rate in 28 joints (CRP)	1.6 ± 1.0	5.2 ± 2.5	6.4 ± 2.5	<0.002	0.099
Swollen joint count	1.0 ± 1.5	11.9 ± 8.8	12.5 ± 9.3	<0.002	0.993
Tender joint count	0.9 ± 1.2	11.5 ± 8.5	12.6 ± 8.5	<0.002	0.904
Visual analog scale	4.6 ± 8.6	21.8 ± 25.8	56.3 ± 37.8	<0.002	0.30
Patient global activity	10.1 ± 9.2	23.6 ± 22.4	55.1 ± 37.9	0.0088	0.027
Evaluator global activity	6.5 ± 4.7	25.1 ± 28.5	42.7 ± 31.1	0.0056	0.200

## Data Availability

The data used to support the findings of this study are included within the article.
